# Clinical Features of Dermatomyositis/Polymyositis with Anti-MDA5 Antibody Positivity

**DOI:** 10.1155/2022/7102480

**Published:** 2022-07-30

**Authors:** Qiuhe Chen, Long Qian

**Affiliations:** Department of Rheumatology and Immunology, The Second Affiliated Hospital of Anhui Medical University, Hefei 230601, China

## Abstract

This paper aims to investigate the clinical and laboratory test characteristics of patients with anti-MDA5 antibody-positive PM/DM by analyzing the clinical characteristics, laboratory test results, and 1-year survival rate of patients with anti-MDA5 antibody-positive PM/DM in polymyositis (PM) and dermatomyositis (DM). To further investigate the impact of positive anti-MDA5 antibodies on the prognosis of PM/DM patients. According to the anti-MDA5 antibody test results, 18 cases with positive anti-MDA5 antibodies were in the positive group and 46 cases with negative anti-MDA5 antibodies were in the negative group. The clinical manifestations, laboratory tests, treatment protocols, and prognostic risk factors were collected for both groups. The chi-square test, Mann–Whitney method, Fisher test, *t*-test, Kaplan–Meier method, and Log-rank test were used for statistical analysis. Anti-MDA5 antibody positivity was more common in patients with DM/CADM. With no statistically significant differences in age and sex ratio between the two groups, The differences in erythrocyte sedimentation rate (ESR), ferritin (Fer), and creatine kinase (CK) levels in the positive group were statistically significant compared with the negative group. Clinically, the positive group was more prone to arthralgia, skin rash, and interstitial pneumonia.

## 1. Introduction

Idiopathic inflammatory myopathies (IIMs) are a group of autoimmune connective tissue diseases that are commonly characterized by an infiltration of inflammatory cells in muscle tissue dominated by T lymphocytes, often involving other organs, such as the skin, joints, lungs, gastrointestinal tract, and heart. Based on muscle symptoms, rash, and histopathological features, IIM was classified into different subgroups, including polymyositis (PM), dermatomyositis (DM), inclusion body myositis (IBM), immune-mediated necrotizing myopathy (immune-mediated necrotizing myopathy (IMNM) and overlapping myositis (with the antisynthetase syndrome, ASS). Limitations of this division are that histopathological features may overlap between subgroups and are poorly specific between individual patients, and isolated features such as inflammation are not specific to IIMs. In addition, the response to treatment and prognosis vary among subgroups due to their different pathogenesis. Therefore, the need to combine histopathological features with clinical and serological data and to include electromyography and muscle biopsy in the classification and diagnosis of IIMs is emphasized, but the methods are cumbersome and patient compliance is poor [1, 2]. Since different subtypes are involved in different clinical processes and respond differently to treatment, the classification of different subgroups of IIMs should better correlate with the underlying disease processes to improve the speed and accuracy of diagnosis, so that patients can receive appropriate treatment and achieve a good prognosis [3, 4].

Compared to the above diagnostic methods, performing myositis-specific autoantibodies (MSAs) tests are painless and convenient, and the clinical phenotypes of different MSAs and PM/DM are closely related, which can help in the early detection of the disease in predicting the clinical course and prognosis of patients. In this study, we investigated the effects of anti-MDA5 antibodies on the clinical characteristics and prognosis of PM/DM patients by comparing and analyzing the basic information, clinical manifestations, laboratory findings, death, the occurrence of complications, and treatment in PM/DM patients in the positive and negative anti-MDA5 antibody groups [5–9].

## 2. Materials and Methods

### 2.1. Subjects and Grouping

Sixty-four patients with a clear diagnosis of PM/DM/clinically amyopathic dermatomyositis (CADM) were collected from 01/2000 to 04/2020 in our hospital. All patients met the diagnostic criteria for PM/DM proposed by Bohan and Peter in 1975 and the modified Sontheimer criteria. (idiopathic inflammatory myopathy, IIM).

This is a group of systemic autoimmune connective tissue diseases, which are mainly divided into dermatomyositis (DM), polymyositis (PM), immune-mediated necrotizing myopathy (IMNM), inclusion body myositis (IBM), and overlap syndrome myositis based on clinical and immunopathological characteristics.

1. Dermatomyositis (DM): typical manifestations are symmetrical muscle weakness, elevated muscle enzymes, and characteristic skin manifestations. There may be antinuclear antibodies (ANA), and some patients have DM-specific autoantibodies, such as anti-Mi-2.
2. Clinically myopathic dermatomyositis (CADM) is a special type: patients have skin manifestations, but lack clinical evidence of muscle involvement.
3. Polymyositis (PM): lack of DM characteristic skin manifestations, muscle weakness, and elevated muscle enzymes. Patients were classified according to whether they were positive for anti-MDA5 antibodies in their autoantibodies, with 18 cases positive for anti-MDA5 antibodies in the positive group and 46 cases negative for anti-MDA5 antibodies in the negative group [10, 11].

### 2.2. Clinical Information

#### 2.2.1. General Data Collection

Basic information of all patients including age and gender, the presence of clinical manifestations such as cough, fever, chest tightness, and shortness of breath, arthralgia, skin rash (mainly Gottron sign and yang-ward rash) before treatment, death, interstitial lung disease (ILD), pulmonary fibrosis, and complications such as interstitial lung disease (ILD), pulmonary fibrosis, infection, and treatment options was collected [3, 12, 13].

#### 2.2.2. Laboratory Tests

Laboratory indicators for the same period included myositis spectrum antibodies, white blood cell (WBC), C-reactive protein (CRP), erythrocyte sedimentation rate (ESR), neutrophil-to-lymphocyte ratio (NLR), ferritin (Fer), creatine kinase (CK), and lactate dehydrogenase (LDH).

### 2.3. Statistical Treatment

SPSS21.0 statistical software was used to analyze and organize the data. Count data were described by the number of cases (percentages), and comparisons between groups were made by the chi-square test or Fisher exact test; measurement data were tested for normality by the Shapiro–Wilk method line data line, and normally distributed measurement data were described by *x* ± *s*, and comparisons between groups were analyzed by *t*-test, nonnormally distributed measurement The data were described by M (P25, P75), and comparisons between groups were analyzed by the nonparametric rank-sum test Mann–Whitney method. The evaluation of patient survival was performed by the Kaplan–Meier method, and median survival and event-free survival time were derived by the log-rank test for single factors. *P* < 0.05 was considered a statistically significant difference [14–16].

## 3. Results

### 3.1. Comparison of General Information between Positive and Negative Groups

With no statistical differences in age and sex ratio between the two groups, it was found that positive anti-MDA5 antibodies were more common in patients with DM/CADM (*P* = 0.006). In terms of clinical manifestations, arthralgia and Gottron's sign were statistically different between the two groups, while the rest of the clinical manifestations and mortality were not different, as shown in Table 1. This revision integrates the entire contents of the clinical data collection into the general data, and at the same time, in the observation index and evaluation index section, the contents of (1) and (2) are exchanged and re-expressed. The title and content have been adjusted in the full text. The biggest adjustment this time is to move the flowchart and the analysis content of the flowchart to the results section to ensure the proper connection of the full text. The results section also changes the order of Table 1, which is easy for readers to understand. In addition, this revision incorporates the content of “Outcome Classification of Cervical Histology LSIL Lesions” into the Outcome Analysis section of the flowchart. Finally, this revision integrates the content of “The predictive value of different HPV E6/E7 mRNA expression on the prognosis of cervical LSIL patients” into the content of the analysis of results in Table 1.

### 3.2. Comparison of Laboratory Test Results between Positive and Negative Groups

The levels of ESR, ferritin, and CK in the positive group were lower than those in the negative group, while the levels of WBC, CRP, NLR, and LDH were not statistically different, as shown in Table 2.

### 3.3. Comparison of Complications between the Positive and Negative Groups

Interstitial pneumonia occurred in 17 patients (94.4%) in the positive group, and its proportion was statistically different (*P* = 0.012) compared with 29 patients (63.0%) in the negative group, as shown in Table 3.

### 3.4. Comparison of Treatment Regimens between Positive and Negative Groups

In the positive group, there were 8 cases of high-dose hormone + immunosuppressant (tacrolimus 3, azathioprine 1, cyclophosphamide 1, azathioprine + cyclophosphamide 2, and cyclosporine 1), 10 cases of low-dose hormone + immunosuppressant (hydroxychloroquine 1, tacrolimus 7, azathioprine 1, and cyclophosphamide 1), and 0 cases of hormone treatment, compared with the negative group. In the negative group, there were 15 cases of high-dose hormone + immunosuppression (6 cases of tacrolimus, 5 cases of cyclophosphamide, 1 case of cyclosporine, and 3 cases of methotrexate), 22 cases of low-dose hormone + immunosuppression (4 cases of hydroxychloroquine, 5 cases of tacrolimus, 5 cases of azathioprine, 4 cases of cyclophosphamide, 1 case of cyclosporine, and 3 cases of methotrexate), and 9 cases of hormone treatment only, and the differences between treatment regimens 2 and 3 were statistically significant (*P* < 0.05) (there was a statistically significant difference between treatment regimens II and III (*P* < 0.05), as shown in Table 4. 10 patients in the positive group with treatment regimen II had statistically significant differences in death (*P* < 0.05), as shown in Table 5.

### 3.5. Analysis of 1-Year Survival between Positive and Negative Groups

The overall 1-year survival rate of the two groups was 94.3%, and the 1-year survival rate of patients in the positive group (76.2%) was lower than that of patients in the negative group (97.4%), and the difference between the two groups was statistically significant (*P* = 0.034), indicating that the negative group had a better prognosis and longer survival time than the positive group, as shown in Table 6, and the survival curves are shown in Figure 1.

## 4. Discussion

An anti-MDA5 antibody is a peptide autoantibody found by Sato et al. in the serum of patients with DM by immunoprecipitation, initially named CADM-140 antibody, and later validated and renamed as an anti-MDA5 antibody. It was found that positive anti-MDA5 antibodies were associated with a high prevalence in patients with DM, especially in CADM patients with no or mild muscle symptoms, and Chen et al. found that nearly half of adult CADM patients had anti-MDA5 antibodies. However, anti-MDA5 antibodies are not only found in adult patients, but Tansley et al. found that anti-MDA5 antibodies were present in 7–24% of adolescent DM patients [17–19]. Recent studies have found a strong association between anti-MDA5 antibody positivity and the clinical manifestations and poor prognosis of DM, an autoimmune disease. In this study, by comparing the general data, laboratory findings of patients with positive and negative anti-MDA5 antibodiesDeaths were analyzed to clarify whether anti-MDA5 antibodies are affected by age, gender, and treatment modality, to reveal common complications and abnormal laboratory test indices in positive patients, and to investigate the effect of positive anti-MDA5 antibodies on cause-specific mortality in middle-aged and elderly PM/DM patients to help in disease prediction diagnosis and prognosis evaluation [20–24].

Related studies have shown that NLR is a classical marker of systemic inflammatory response. You-Jung et al. found that high NLR (>4.775) was significantly associated with patient survival and acute interstitial pneumonia. Therefore, it is speculated that NLR level may be a simple and economic prognostic indicator in patients with polymyositis/dermatomyositis. However, we have not found a correlation between NLR values and the presence or absence of positive anti-MDA5 antibodies and patient mortality (*P* > 0.05), suggesting that NLR is not an independent influence on mortality in patients with PM/DM-ILD. The combined carcinoembryonic antigen (CEA) and Ferritin levels were found to reflect the severity of anti-MDA5 antibody-positive DM combined with ILD. The differences in ESR levels, Ferritin levels, and CK levels between the two groups were analyzed to be statistically significant. Therefore, it was hypothesized that the combination of these three laboratory tests could be used to predict and diagnose the severity of patients with anti-MDA5 antibody-positive PM/DM.ILD was found to be one of the most common systemic complications of IIM, and ILD associated with DM, especially in patients with anti-MDA5 antibody-positive CADM, has a rapid progression and poor prognosis. In many retrospective cohort studies, the specificity of rapidly progressive ILD in PM/DM patients was 86% and the sensitivity was 77%, and among patients with DM, PM, or PM/DM-related ILD, anti-MDA5-positive patients had the worst prognosis, with almost half of them dying within 6 months of diagnosis. Thus, there are many reports that anti-MDA5 antibody positivity is closely associated with ILD and suggests a poor prognosis, but there are fewer reports on the overall survival of anti-MDA5 antibody-positive PM/DM patients. In this study, we concluded that there was a significant correlation between ILD and anti-MDA5 antibody positivity (*P* = 0.012) and that patients with anti-MDA5 antibody-positive PM/DM were more likely to have comorbid ILD, but the difference of 3 deaths (16.7%) in the positive group versus 1 death (2.2%) in the negative group was not statistically significant based on the follow-up results. By calculating the death of patients in the follow-up results only, it was obvious that there were time limitations and missing follow-up values, so a survival curve analysis was performed and it was found that the overall 1-year survival rate was 94.3% between the two groups of 64 patients who were anti-MDA5 positive and anti-MDA5 negative, and the 1-year survival rate of anti-MDA5 positive patients (76.2%) was lower than that of anti-MDA5 antibody negative patients (97.4%). The difference between the two groups was statistically significant (*P* = 0.034), suggesting that patient prognosis analysis needs to be overlaid with a focus on all time points rather than specific time points and that anti-MDA5 antibody positivity is strongly associated with poor prognosis throughout the course of combined ILD in patients with PM/DM. For treatment options in patients with PM/DM-ILD, there is evidence that immunosuppressive therapy is effective in the combination of acute progressive ILD in patients with anti-MDA5 antibody-positive CADM. However, Mimori et al. found that effective immunosuppressive combination therapy using high-dose glucocorticoids, calcium-modulated neurophosphatase inhibitors, and cyclophosphamide should be considered as induction therapy for acutely progressive ILD, which is poorly effective and has a poor prognosis for patients with anti-MDA5 antibody-positive CADM who do not develop ILD. There is no evidence-based treatment for PM/DM-ILD [25, 26].

There are several limitations in this study. First, as a retrospective case study, the total number of cases collected was small, and some of the follow-up cases were excluded due to incomplete information. Second, we collected PM/DM patients all from the same hospital in the same region, which has some regional limitations. In addition, patients' treatment decisions were dependent on the primary care physician and did not use a consistent protocol, resulting in the inability to correlate the relationship between death and treatment protocol. In addition, due to the small number of included indicators, the multivariate analysis could not be performed and no optimized predictive and diagnostic indicators were provided [27–29]. Through literature research, relevant indicators and early clinical manifestations that may assist in the diagnosis and prognostic outcome of patients with anti-MDA5 antibody-positive PM/DM were identified. Through serum marker mining, interleukin 6 and cytokeratin 19 fragments were found to be associated with anti-MDA5 interleukin-18 is involved in the development of acute interstitial pneumonia and may assist in the diagnosis of patients with anti-MDA5 antibody-positive PM/DM. Routine blood tests and clinical manifestations revealed that CD3+CD4+ T cell levels and the development of hypoxemia at the beginning of the disease were positively correlated with mortality in patients with anti-MDA5 antibody-positive dermatomyositis, which may indicate a poor prognosis. Therefore, more prospective studies incorporating more laboratory examination indices and clinical manifestations assessment are needed to further understand the course of disease activity and prognosis in patients with anti-MDA5 antibody-positive PM/DM.

In conclusion, it was found that anti-MDA5 antibody positivity is more common in patients with DM and that anti-MDA5 antibody positivity is more likely to be combined with interstitial pneumonia and poorer survival than anti-MDA5 antibody negative patients, with differences in ESR, Ferritin, and CK levels between the positive and negative groups. Although the diagnosis of PM/DM may be influenced by different factors, such as the early stage of the disease, the need for a correct diagnosis, and the overall experience of the clinician.

## Figures and Tables

**Figure 1:** Survival curves of the positive and negative groups.

**Table 1:** Comparison of each clinical information between positive and negative groups*n* (%), *x* ± *s*.

	Positive group (*n* = 18)	Negative group (*n* = 46)	*χ * ^2^/*t*/*Z*	*P*
Sex			3.677^*∗*^	0.055
Men	11 (61.1)	16 (34.8)		
Women	7 (38.9)	30 (65.2)		
Age (years)	52	51	0.398^#^	0.692
Diagnosis				
DM + CADM	17 (94.4)	27 (58.7)	7.696^*∗*^	0.006
PM	1 (5.6)	19 (41.3)		
Cough	9 (50.0)	20 (43.5)	0.222^*∗*^	0.637
Chest tightness and shortness of breath	11 (61.1)	21 (45.7)	1.237^*∗*^	0.266
Joint pain	12 (66.7)	16 (34.8)	5.344^*∗*^	0.021
Gottron sign	10 (55.6)	9 (19.6)	8.028^*∗*^	0.005
Sunburn rash	6 (33.3)	8 (17.4)	1.104^*∗*^	0.293
Rash				
Others	1 (5.6)	10 (21.7)	1.379^*∗*^	0.240
None	1 (5.6)	19 (41.3)	7696^*∗*^	0.006
Death	3 (16.7)	1 (2.2)	2.494^*∗*^	0.114

*Note.* ^*∗*^Chi-square test; ^#^*t*-test.

**Table 2:** Comparison of laboratory test results between positive and negative groups *M* (P25, P75).

	Positive group (*n* = 18)	Negative group (*n* = 46)	*χ * ^2^/*t*/*Z*	*P*
WBC ( ^*∗*^109/L)	8.025 (5.689, 10.033)	6.000 (4.438, 10.300)	−1.755^Δ^	0.079
CRP (mg/L)	4.800 (1.681, 22.000)	7.533 (2.993, 12.200)	−0.274^Δ^	0.784
ESR (mm/1h)	16.000 (6.500, 38.000)	33.000 (18.500, 46.750)	−2.413^Δ^	0.016
NLR (%)	4.063 (2.890, 6.427)	4.117 (3.005, 7.457)	−0.687^Δ^	0.492
Ferritin (ng/ml)	266.100 (129.500, 510.850)	1133.000 (685.000, 2616.000)	−3.904^Δ^	0.000
CK (U/L)	91.000 (47.000, 369.000)	537.500 (67.500, 2013.500)	−2.330^Δ^	0.020
LDH (U/L)	327.000 (222.000, 464.000)	315.000 (253.000, 469.500)	−0.066^Δ^	0.948

*Note.* Mann–Whitney method.

**Table 3:** Comparison of complications between the positive and negative groups (*n* (%)).

	Positive group (*n* = 18)	Negative group (*n* = 46)	*χ * ^2^	*P*
Interstitial pneumonia	17 (94.4)	29 (63.0)	6.311^*∗*^	0.012
Pulmonary fibrosis	0 (0.0)	6 (13.0)	1.283^*∗*^	0.257
Infection	7 (38.9)	11 (23.9)	1.435^*∗*^	0.231

*Note.* ^*∗*^Chi-square test.

**Table 4:** Comparison of treatment regimens between the positive and negative groups (*n* (%)).

	Positive anti-MDA5 antibody (*n* = 18)	Negative anti-MDA5 antibody (*n* = 46)	*χ * ^2^	*P*
Treatment 1	8 (44.4)	15 (32.6)	0.222^*∗*^	0.637
Treatment 2	10 (55.6)	22 (47.8)	4.500^*∗*^	0.034
Treatment 3	0	9 (19.6)	9.000^*∗*^	0.002

*Note.* ^*∗*^Chi-square test; Treatment 1: methylprednisolone ≥ 60 mg/d + immunosuppression; Treatment 2: methylprednisolone < 60 mg/d (or oral equivalent prednisone) + immunosuppression; Treatment 3: hormones only without combined immunosuppression.

**Table 5:** Prognosis analysis of 18 patients with positive anti-MDA5 antibodies with different treatment modalities (*n* (%)).

Treatment modality	Survival (*n* = 15)	Death (*n* = 3)	*χ * ^2^	*P*
Treatment 1	6 (40.0)	2 (66.7)	2.000^*∗*^	0.157
Treatment 2	9 (60.0)	1 (33.3)	6.400^*∗*^	0.011
Treatment 3	0	0	—	—

*Note.* ^*∗*^Chi-square test; Treatment 1: methylprednisolone ≥ 60 mg/d + immunosuppression; Treatment 2: methylprednisolone < 60 mg/d (or oral equivalent prednisone) + immunosuppression; Treatment 3: hormones only without combined immunosuppression.

**Table 6:** K-M survival analysis in the positive and negative groups.

	*n*	1-year OS (%)	*χ * ^2^	*P* value	Median OS time (months)		
					Estimated value	95% CI	
						Lower limit	Upper limit
Overall	64	94.3			267.916	244.914	290.917
Anti-MDA5 antibody			4.503	0.034			
Negative	46	97.4			284.641	270.404	298.878
Positive	18	76.2			31.833	25.647	38.020

## Data Availability

The experimental data used to support the findings of this study are available from the corresponding author upon request.
